# Complete Healing After Umbilical Mesenchymal Stem Cell-Derived Exosome Therapy For a Refractory Complex Anal Fistula

**DOI:** 10.7759/cureus.104324

**Published:** 2026-02-26

**Authors:** N Cigdem Arslan, Ilknur Erenler, Erdal Karaoz

**Affiliations:** 1 General Surgery, Istanbul Health and Technology University, Istanbul, TUR; 2 General and Colorectal Surgery, Private Clinic, Istanbul, TUR; 3 Histology and Embryology, IIstinye University, Istanbul, TUR; 4 Center for Regenerative Medicine and Stem Cell Research and Manufacturing (LivMedCell), Liv Hospital Ulus, Istanbul, TUR

**Keywords:** anal fistula, complex wound, exosome therapy, recurrent fistula, stem cell

## Abstract

Complex anal fistulas pose a persistent challenge due to high recurrence and the risk of continence impairment. While sphincter-sparing techniques exist, outcomes are variable in refractory disease. Mesenchymal stromal cell (MSC) therapies show promise but face logistical barriers, prompting interest in acellular exosome-based approaches. We report a 45-year-old woman with a complex anterior anal fistula refractory to multiple surgeries, including two endoanal advancement flaps, complicated by new-onset flatus incontinence. Following the second endoanal advancement flap, the patient's Cleveland Clinic Continence Score (CCIS) was 10, and the Quality of Life in Patients with Anal Fistula Questionnaire (QoLAF-Q) score was 51. A two-stage salvage strategy was undertaken: meticulous curettage and closure of the internal opening, followed by local administration of MSC-derived exosomes at baseline and three weeks. Significant wound reduction was observed, progressing to complete epithelialization within two weeks after the second exosome application. At six months after combined surgical intervention and exosome therapy, CCIS and QoLAF-Q scores improved to 0 and 28, respectively, indicating full restoration of continence and a marked improvement in quality of life.

This case suggests that local exosome therapy, used as an adjunct to careful surgical preparation, may support healing and functional recovery in refractory complex anal fistulas. Controlled studies with standardized protocols are warranted to define efficacy, dosing, and durability.

## Introduction

Complex anal fistulas represent a significant clinical challenge in anorectal surgery due to the high risk of recurrence and functional compromise [1]. Management is defined by an inherent dichotomy between achieving definitive healing and preserving anal continence [2]. This difficult trade-off has led to the development of numerous sphincter-preserving techniques, yet their efficacy remains highly variable, particularly in refractory cases [3].

Among established sphincter-sparing procedures for cryptoglandular complex fistulas, the endoanal advancement flap (EAF) reports pooled failure rates of 20-25% with continence disturbance rates ranging between 7 and 10% [3,4]. Newer, less invasive methods, such as fistula laser closure, typically preserve function better, with reported continence disturbance rates as low as 1% in a recent meta-analysis; however, this safety comes at the cost of high failure rates reported at 33% [1,5]. The need for salvage therapies is magnified in especially difficult presentations, such as complex recurrent fistulas, cases involving the anterior sphincter in women, and perianal Crohn’s disease [6].

Considering the suboptimal outcomes of conventional surgery, particularly in refractory disease, mesenchymal stromal cells (MSCs) emerged as a promising regenerative alternative, leveraging their trophic, anti-inflammatory, and immunomodulatory properties [6]. For Crohn’s fistulas, MSCs, specifically allogeneic adipose-derived stem cells (Cx601), demonstrated superior results over placebo, achieving combined remission in 50% of patients at 24 weeks versus 34% in the placebo group (p=0.024) in the landmark ADMIRE trial [7]. A recent meta-analysis including Crohn’s and cryptoglandular (non-Crohn’s) complex fistulas reported the pooled healing rate for autologous MSC therapy as 58.4% (48.3-68.5%) [8].

Despite this therapeutic success, the widespread implementation of MSC therapy is hindered by infrastructural challenges related to cell sourcing, expansion, and associated regulatory complexities [9]. Consequently, research has shifted towards extracellular vesicles (exosomes), which are shed by MSCs and carry the key regenerative functionality (secretome) but offer the logistical advantage of an "off the shelf" product [9]. Recent preliminary studies have explored the use of MSC-derived exosome therapy in both Crohn’s and non-Crohn’s complex anal fistulas, but available data in the literature remain very limited [10-12].

We present a case of a woman with an anterior anal fistula who had functional deterioration following multiple failed surgical attempts. This case report illustrates the potential of localized exosome therapy to achieve complete anatomical healing and functional restoration in complex fistulas.

## Case presentation

Patient background

The patient is a 45-year-old woman with a four-year history of recurrent perianal fistula. Clinical examination and imaging confirmed the diagnosis of a complex anterior anal fistula. The external opening was located in the left anterolateral perineum (1 o'clock in lithotomy position), approximately 6-7 cm from the anal verge. The fistula tract coursed superiorly and medially to an internal opening at the anterior midline of the anal canal. She had two colonoscopies with no signs of inflammatory bowel disease.

Previous surgeries

Between 2021 and 2024, she initially underwent multiple incision and drainage procedures for recurrent abscesses, followed by two separate attempts at fistula tract closure using a laser, both of which failed. The patient subsequently underwent two EAFs. The first procedure failed with early recurrence at three months (Figure 1). The second EAF, performed in February 2025 in our institution, resulted in complete flap dehiscence and fecal leakage on the fourth postoperative day. Following the second flap failure, a loose seton was placed to control sepsis and manage chronic drainage (Figure 2a). At this point, the patient reported new‑onset flatus incontinence. The seton was removed two weeks later.

**Figure 1:** Axial T2-weighted fat-suppressed images demonstrate the recurrent anal fistula after the patient’s third surgery. The white arrows indicate the internal opening at the anal canal, and the yellow arrows mark the external opening in the left anterior perineal skin.

**Figure 2:** Before exosome therapy a) Immediate placement of a loose seton after failure of the second endoanal advancement flap, b) Appearance at 3-month follow-up, showing a persistent defect that has not decreased in size and has evolved into a chronic wound.

Exosome therapy rationale

Between March and May 2025, the patient was closely observed with a large persistent defect that did not appear to be getting smaller (Figure 2b). The flatus incontinence has persisted. The Quality of Life in Patients with Anal Fistula Questionnaire score (QoLAF-Q) [13] was 51 (range 14-70), revealing a high impact on QoL, and the Cleveland Clinic Incontinence Score (CCIS)[14] was 10 (range 0-20). Given the patient's extensive history of four failed surgical interventions and the development of new-onset incontinence, a decision was made to employ a novel therapeutic approach. The persistence of the fistula indicated a biological failure to heal that was unlikely to be resolved by another purely mechanical procedure. Therefore, an exosome-based therapy was decided as a biologic adjunct to meticulous surgical debridement with the patient’s informed consent.

Exosome production and quality processes

The MSCs used in this study were obtained from LivMedCell - licensed and approved by the Turkish Ministry of Health, produced under Good Manufacturing Practice (GMP) conditions, and maintained at Liv Hospital Ulus, as previously described [15]. For exosome production, the following procedure was followed:

WJ-MSC-derived exosomes are obtained by isolating from mesenchymal stem cells brought to passage 4 (P4). Mesenchymal stem cells are thawed at P3. After the cells are centrifuged, they are diluted with culture medium (NutriStem), seeded, and placed in an incubator at 37 °C containing 5% CO₂. When the cell density reaches 60-70% confluency, the medium on the cells is removed and washed with PBS. DMEM F12 medium is added on the cells and incubated for 24-48 hours at 37 °C containing 5% CO₂. After incubation, culture supernatants are collected in Falcon tubes. The supernatant is centrifuged sequentially at increasing speeds to remove large dead cells and large cell debris. The pellet is removed, and the supernatant is used for the next step. The supernatant is passed through a syringe filter and transferred into an ultracentrifuge tube. The supernatant is centrifuged at 10,000 g for 60 min and 110,000 g for 120 min. At this stage, the pellet is used. The pellet is diluted and centrifuged at 110,000 g for 120 min. The supernatant is removed. The exosome pellet is diluted with physiological saline or dPBS.

Nanoparticle tracking analysis (NTA) (Malvern Panalytical NanoSight NS300, UK) and Flow Cytometers (BD FACSCanto™ II) are used for characterization. The particle amount and size of the exosome samples are determined by the NTA device. The positivity of CD81, CD9 and CD63 markers of exosome samples is determined by flow cytometry using the Tetraspanin Exo-Flow Capture Kit (System Biosciences). Product safety is ensured by performing the mycoplasma test, Gram staining, and endotoxin test on exosome samples. The final exosome preparation was characterized by particle concentration and total protein content prior to administration, with sterility and endotoxin testing performed according to institutional GMP protocols. The injectate was prepared immediately before use under sterile conditions, and its clinical application was conducted within the institutional regulatory/ethics framework after obtaining written informed consent from the patient.

Surgical procedure and intervention

The surgical technique was performed as a two-stage application, designed to prepare the wound bed and then support the regenerative process. The procedure drew parallels from surgical protocols used in cellular therapy trials [16].

Step 1 (02-June-2025)

Initial debridement and exosome application: Under local anesthesia, the patient was placed in the left decubitus position. The fistula tract was meticulously debrided using curettage to remove all granulation and fibrotic tissue, creating a fresh wound bed. The internal opening of the fistula was closed with absorbable sutures. The first dose of the exosome product (5 ml, 1.0×10¹⁰ particles measured by NTA) was injected directly into the walls of the fistula tract and the surrounding tissue (Figure 3).

**Figure 3:** Debridement and exosome therapy a) Sharp debridement with undermining of devitalized tissue and epithelialized wound edges, b) Closure of the internal opening, c–f) Exosome injections delivered both deep and superficial along the wound.

Step 2 (23-June-2025)

Second application: Three weeks after the initial procedure, the wound showed significant signs of healthy granulation and reduction of more than 50% in size (Figure 4a). A second application of the exosome product (5 ml, 1.0×10¹⁰ particles measured by NTA) was administered to the wound to provide continued regenerative stimulus.

**Figure 4:** The healing process a) Three weeks after the first exosome application, b) One week after the second exosome application, c) Complete healing at three weeks after second exosome application, d-e) Axial contrast‑enhanced T1 images at six months magnetic resonance examination demonstrates no residual tract or collection, intersphincteric and ischioanal fat planes are restored, and the internal opening appears closed with scar tissue, findings consistent with a healed anal fistula.

Outcome assessment and follow-up

The primary endpoints for treatment success were defined as follows.

Complete Healing

Full epithelialization of the external opening with no evidence of drainage, either spontaneously or upon gentle compression of the tract, was confirmed with MRI at six months.

Improvement of Quality of Life

Resolution of fistula symptoms and incontinence measured by QoLAF-Q and CCIS. The QoLAF questionnaire, designed to assess health-related quality of life specifically in anal fistulas, comprises physical and biopsychosocial impact domains, with a summed score from 14 to 70 (14 = zero impact, 15-28 = limited, 29-42 = moderate, 43-56 = high, 57-70 = very high impact) [13]. The CCIS, a validated five-item measure of stool and gas incontinence (type and frequency) plus pad use and lifestyle alteration, yields a total score from 0 (perfect continence) to 20 (complete incontinence) [14].

Clinical assessments were performed at one week and two weeks post-intervention in outpatient clinic. A definitive follow-up was conducted at six months, which included both a clinical examination and a radiological assessment to confirm the absence of any persistent or recurrent fistula tract or fluid collection.

Results

A favorable clinical and functional outcome was observed following the salvage surgical intervention with exosome therapy.

Three Week Post-intervention

At the three-week follow-up after the first application, the external wound had reduced in size by approximately 50% (Figure 4a). The patient reported a significant decrease in discharge and perianal discomfort.

Complete Healing

Following the second exosome application, the wound continued to show progressive closure (Figure 4b). Within three weeks of the second procedure, complete clinical healing was achieved, with full epithelialization of the external opening and no evidence of drainage upon gentle compression (Figure 4c).

Six-Month Follow-Up

At the definitive six-month follow-up, the patient remained fully healed. Both clinical examination and radiological imaging confirmed the complete and sustained closure of the fistula tract, with no signs of abscess, fluid collection, or recurrence (Figure 4d). In November 2025, six months after the first exosome application, MRI confirmed complete clinical healing (Figures 4e, 4f). The QoLAF-Q score was 51 after the second EAF and improved to 28-driven predominantly by psychosocial and sexual domain burdens, which had been the patient’s highest-scoring areas. The CCIS was 10 after the second EAF and improved to 0 at 6 months, indicating complete restoration of continence.

Intervention adherence, tolerability, and patient perspective

Beyond the anatomical success, the functional outcome was equally significant. The patient expressed profound satisfaction with the outcome, highlighting the dramatic positive impact on her quality of life. The flatus incontinence resolved completely following fistula closure. The intervention was very well-tolerated, with no adverse events reported.

## Discussion

In this case of a highly refractory complex anterior anal fistula, meticulous surgical debridement combined with local exosome application was associated with rapid and sustained healing. Notably, sphincter function returned to baseline, with resolution of treatment-emergent incontinence. While causality cannot be assigned to exosomes alone, given the concurrent surgical measures, these findings suggest that an acellular, regenerative approach may have a supportive role in difficult-to-heal fistula biology.

The patient's history represents a "worst-case scenario" for anal fistula surgery. Several factors likely contributed to the repeated failures. The anterior location of the fistula in a female patient, a long and established tract, and a history of recurrence are all well-recognized risk factors for poor surgical outcomes [1]. The failure of two EAFs is consistent with literature showing that success rates for this procedure can be as low as 37% in complex cases [17]. These mechanical repairs rely on healthy, well-vascularized tissue for success, a condition often absent in the setting of chronic inflammation and scarring. This underscores the need for therapies that can improve compromised tissue features in such surgical sites without functional trade-offs.

We hypothesize that exosome therapy succeeded where surgery failed by addressing the underlying biological problem: a local tissue environment locked in a state of chronic, non-healing inflammation. Drawing from the known paracrine functions of MSCs, exosomes likely delivered a complex secretome that fundamentally altered the local tissue biology [9,18]. This biological payload is thought to exert several key effects: (i) Immunomodulation, suppressing the chronic pro-inflammatory state that prevents healing; (ii) Anti-fibrosis, inhibiting the excessive scarring that characterizes refractory fistulas; (iii) Pro-regeneration: Stimulating angiogenesis (new blood vessel formation) and promoting the migration and proliferation of epithelial cells. This biological modulation is a critical adjunct to the meticulous surgical debridement, which creates a receptive wound bed but cannot, on its own, overcome the inherent biological failure-to-heal in such refractory cases. Instead of simply closing a defect with scarred tissue, the regenerative approach aims to foster an environment conducive to organized, functional tissue repair.

The healing observed in this case aligns with the most successful outcomes reported for live MSC therapies. The efficacy of MSCs for complex fistulas has been consistently demonstrated, with major trials and cohort studies reporting healing or remission rates in the 50% to 67% range [7,16]. The pivotal ADMIRE CD trial reported a 50% combined remission rate with allogeneic adipose-derived MSCs, which was significantly higher than the 34% rate observed in the placebo group [7]. Recent meta-analyses have consistently confirmed that cell-based therapies are superior to placebo or conventional treatments [19,20]. As an acellular, "off-the-shelf" product, it circumvents many of the logistical and biological challenges associated with viable cell therapies. These characteristics suggest exosome therapy has the potential to overcome the logistical barriers of complex cell culture infrastructure, concerns about cell viability from manufacturing to administration, limited shelf-life, and the potential for alloimmunity [9].

The literature on exosome therapy for anal fistulas is limited. Small studies in Crohn-associated fistulas have reported encouraging safety and healing outcomes [11,12]. As the present patient did not have Crohn’s disease, interpretation of the treatment effect should rely mainly on non-Crohn data. In non-Crohn fistulas, Pak et al. [10] reported a 45% healing rate in refractory cases. They derived exosomes from placental MSCs and administered 25 billion particles per tract (0.5×1010 particles/mL, 5 mL injectables) weekly, three times. In our case, we administered umbilical MSC-derived 10 billion particles twice, and the duration between sessions was three weeks. The healing was confirmed with both clinical and radiological assessment in both studies. Pak’s study reported improvement in QoL scores; however, it was unclear what scale or questionnaire was used or if it was specific to anal fistula or continence [10]. A critical aspect of our case was the restoration of sphincter function with the resolution of flatus incontinence and improved QoL scores. The functional result is consistent with findings from MSC trials, where improvements in incontinence scores have also been reported [16]. This outcome can contribute to the goal in complex fistula management: complete anatomical healing with full functional restoration.

Limitations and future directions

The primary limitation of this report is that it describes the outcome of a single case with only six months’ follow-up. The clear path forward requires rigorous scientific validation. Prospective, randomized controlled trials with longer follow-up durations are essential to confirm these findings. Future trials must be designed not only to validate efficacy but also to rigorously define key therapeutic parameters, such as the optimal exosome concentration, the necessity of single versus multiple applications, and the long-term durability of the regenerative effect compared directly to viable MSCs. In this case, debridement and closure of the internal opening were performed alongside exosome therapy. Healing cannot be attributed solely to exosome therapy, as concomitant internal opening closure and possible imaging interpretation bias may have contributed to the outcome. Therefore, attributing complete healing solely to exosomes is not justified. Exosomes should be considered an adjunctive, healing-promoting factor rather than the exclusive driver of the outcome. The fact that one of the authors is an employee of the company providing the exosomes represents a potential conflict of interest and should be taken into account when interpreting the results.

## Conclusions

Local administration of umbilical mesenchymal stem cell-derived exosomes, combined with meticulous surgical preparation, may offer a supportive role in the healing of refractory complex anal fistulas. In this case, rapid wound closure and restoration of continence were observed, suggesting potential benefits of exosome therapy as an adjunct. However, these findings are limited to a single patient and short-term follow-up. Larger, controlled studies are needed to clarify the efficacy, safety, and long-term outcomes of this approach.
